The article "Stereotactic Surgery of Parkinson's Disease with Magnetic Resonance Imaging under Three-Dimensional Mark Point Positioning Algorithm" was published in 2022. Journal: Contrast Media Mol Imaging.

# Stereotactic Surgery of Parkinson's Disease with Magnetic Resonance Imaging under Three-Dimensional Mark Point Positioning Algorithm

**DOI:** 10.1155/2022/9383982

**Published:** 2022-06-26

**Authors:** Yuan Jia, Zengguang Wang, Xiang Sun, Yipin Zhou

**Affiliations:** ^1^Department of Neurosurgery, Tianjin Third Central Hospital, Tianjin 300170, China; ^2^Department of Neurosurgery, Tianjin Medical University General Hospital, Tianjin 300052, China

## Abstract

This research aimed to study the application of magnetic resonance imaging (MRI) under three-dimensional mark point positioning algorithm in stereotactic surgery for Parkinson's disease (PD) and improve clinical treatment effect. Eighty patients with PD in Tianjin Medical University General Hospital were selected as the research objects and randomly divided into two groups. The three-dimensional mark point positioning algorithm was applied to perform feature positioning on the MRI images of PD patients, and the international unified Parkinson's disease rating scale (UPDRS) was assessed before and after single-target surgery of the two groups. There was a significant difference in the postoperative treatment effect between the two groups compared with the preoperative one (*P* < 0.05). Among the patients in the observation group, 37 cases were marked as markedly effective, accounting for 92.5% of the total group; 1 case was ineffective and 2 cases were improved, accounting for 2.5% and 5%, respectively. In the control group, 35, 2, and 3 cases were assessed as markedly effective, ineffective, and improved, accounting for 87.5%, 5%, and 7.5%, respectively. The overall curative effect of the observation group was better than that of the control group, and the difference was significant (*P* < 0.05). The MRI manifestations of PD patients were diversified. MRI under the three-dimensional mark point positioning algorithm had a high value for the stereotactic treatment of PD patients, which was beneficial to the clinical surgery.

## 1. Introduction

Parkinson's disease (PD) is also called paralysis agitans, which is a neurodegenerative disease with relatively insidious onset and slow course [1, 2]. Most PD patients are sporadic cases, and a small number of patients with the family history account for 10%. The pathological mechanism of PD mainly lies in glial cell proliferation in different degrees of the substantia nigra pars compacta with dopamine, and the loss of some neurons. However, how this pathology causes PD exactly is still not very clear. The degeneration and death of the neurons need to be further explored, and other reasons such as aging, environmental factors, genetics, and oxidative stress have not yet been clearly known at current [3, 4]. For the population who are attacked by PD at the age of 60 years, relevant data show that there is a certain connection between the disease and aging. However, there is no such a trend in the 65-year-old group, and the morbidity is not high in the 65-year-olds. Therefore, more research is needed on how the neurons of PD patients change [5–7]. The clinical diagnosis of PD mainly relies on symptoms, signs, routine blood sample examinations, medical history, and so on [8]. In the examination of head, magnetic resonance imaging (MRI) and computerized tomography (CT) show no characteristic changes [9]. At present, there is no cure for PD, and the main treatment method is a combination of drugs and surgery. Stereotactic surgery is a method for the treatment of PD [10]. With the rapid development of imaging and neuroelectrophysiology, the use of brain stereotaxic technology to treat PD has become an important treatment method. Stereotactic surgery is safe and effective for PD, and the precise positioning of the target can improve the surgical efficacy and reduce complications.

The article "Stereotactic Surgery of Parkinson's Disease with Magnetic Resonance Imaging under Three-Dimensional Mark Point Positioning Algorithm" was published in 2022. Journal: Contrast Media Mol Imaging.

The motor system of PD patients is abnormal, and the lack of dopamine in the brain causes the dysfunction of cortex-striatum-cortex circuits. How the network with the complex process works and how it performs abnormally are still uncertain. At present, resting-state functional MRI has been used in the research of PD pathology and has shown certain effects. MRI can locate in multiple directions and has high resolution for soft tissues, so that it is widely used for the diagnosis of many diseases clinically [11, 12]. MRI would lead to fewer complications in stereotactic surgery, with less loss and a relatively simpler method [13, 14]. Examination results of MRI can be observed at multiple angles, multiple slices, and multiple directions. The computer system can convert the anatomical mark points into coordinate values, eliminating measurement errors, and can display the morphological structure of the soft tissues of the craniofacial region clearly without radiation. Although MRI can clearly show the structure of the brain tissues, there are relatively few studies on MRI in examining the brain of PD patients [15, 16]. In the clinical practice, there are differences in the position of the two-dimensional image displayed, and the left and right of the anatomical image cannot overlap well, so there is the distortion in image. This also causes error in a certain degree in the diagnosis, resulting in misdiagnosis and missed diagnosis. The two-dimensional image cannot fully show the real anatomy, and the detection result is not correct enough [17]. Three-dimensional imaging in MRI images can clearly show the exact anatomical positioning, display the measurement of the image accurately, and locate the lesion on the three-dimensional brain image of the patients clearly [18, 19].

The article "Stereotactic Surgery of Parkinson's Disease with Magnetic Resonance Imaging under Three-Dimensional Mark Point Positioning Algorithm" was published in 2022. Journal: Contrast Media Mol Imaging.

In the case of clear 3D MRI images, this study constructed a method for locating anatomical markers in the brain, combined with the accurate positioning of surgical targets, which provided a basis for the development of single-scan MRI image parameters and improved surgical efficacy, thus segmenting MRI images, analyzing the characteristics of PD patients from different directions, reducing the incidence of patient complications, and improving the accuracy of surgery.

## 2. Materials and Methods

### 2.1. Research Object

Retrospective analysis of PD patients in Tianjin Medical University General Hospital was made, and those patients were chosen as the research objects. The modern multifunctional video therapy equipment and high-precision brain stereotaxic instrument were used to treat the PD patients who joined the study. 40 patients who underwent three-dimensional mark point positioning surgery were included in the observation group. The age of the patients was 42 ± 72 years with an average age of 51.23 ± 3.24 years, and the course of disease was (11 ± 7). 16 patients out of them had the PD of tremor type, 9 patients had the tetanic PD, and 15 patients had the mixed PD. Another 40 patients in the control group received ordinary surgical treatment. They aged 41 ± 69 years with an average age of 49.23 ± 2.67 years and course of disease of (12 ± 4). 19 of them suffered from tremor PD, 11 patients had the tetanic type, and 10 patients were classified into the mixed type. This study had been approved by ethics committee of hospital, and all the study objects and their families were informed and voluntarily agreed to participate in this study.

The following inclusion criteria were formulated: All study objects were evaluated by experienced neurologists using the unified Parkinson's disease rating scale (UPDRS). The patients offered complete general clinical information. They met the treatment indications and had not interrupted all treatment in the hospital. All the objects self-cooperated with the diagnosis and treatment.

Exclusion criteria were as follows: The patients had language communication disorders, serious diseases like organic diseases of the hematopoietic system, or mental illnesses. Patients had a poor compliance in the treatment. Patients stopped treatment for some cause. Patients had systemic infections or brain diseases in other parts of the body.

### 2.2. MRI Image Acquisition Method

The patients stopped taking levodopa drugs 1 day before the surgery. On the day of the surgery, a stereotactic frame was laid down on the patient's head, and a high-resolution MRI examination was made. For functional positioning, the CRW stereotaxic system utilized was the Leksell system of Elekta AB, Sweden. Brain MRI was performed with 1.5T magnetic resonance machine by Signa, GE Corporation. The receiving coil was an abdominal phased array winding coil, while the radio frequency transmitting coil was a body coil. The sagittal and axial planes were selected for the positioning of the target point under direct vision. The scanning plane was required to be parallel to the anterior commissure-posterior commissure (AC-PC). The coordinates of the target nuclei were located with the midpoint of AC-PC as the original point, *X* = ±10–±13 mm, *Y* = −1 to −2 mm, and *Z* = −2 to −6 mm. The selected conventional coronal and sagittal parameters were as follows. Time of repetition (TR)/time of echo (TE) = (3500–3800) ms/130 ms; for T2WI signal, fat saturation fast recovery fast spin echo (fs FRFSE) was *X*, number of excitations (NEX) = 2–4, the field of view (FOV) = 26. For the sectional spin echo-echo planar imaging (SE-EPI) sequence of diffusion-weighted imaging (DWI), *b* = 700, TR/TE = 4000 ms/73 ms. For the cross-sectional T1WI signal, fat-saturated fast-spin echo (fs FSE) was XL, TR/TE = 400 ms/8 ms, NEX = 2, and FOV = 32. For the cross-sectional T2WI signal, fs FRFSE was XL, TR/TE = 4000 ms/130 ms, NEX = 4, and FOV = 32.

The article "Stereotactic Surgery of Parkinson's Disease with Magnetic Resonance Imaging under Three-Dimensional Mark Point Positioning Algorithm" was published in 2022. Journal: Contrast Media Mol Imaging.

### 2.3. Mark Point Behavior Algorithm

Directed against digital image algorithm for straight line and circular feature detection, image mark point algorithm has been applied in a lot of research worldwide. For straight line features, Paul Hough proposed a transformation method to detect straight lines in binary images. If the variable XY was regarded as a constant, the linear equation in Figure 1(a) was transformed into the parameter space. Then, it was transformed again into a cluster of sinusoids in the parameter space, as shown in Figure 1(b). The edge points of the binary image can be adopted to determine the straight-line equation, which was that the Hough transform was used to detect the straight line.

For the detection of circular mark points, the algorithm was introduced and extended to detect circles, ellipses, and parabolic curves with analytical expression *f* (*x*, *y*) according to the equations. It was assumed that the center of the circle was *O* (*a*, *b*) and the radius was *r*, and the detection of the circular mark points was carried out in the discretized space. The three-dimensional accumulation array *A* (*a*, *b*, *r*) was established, and after any point (*x*_*i*_*, y*_*i*_) on the circumference in the image space was transformed into the parameter space, the corresponding value of *r* could be computed with the changes of center of the circle in the parameters. It was accumulated on point *A*, and finally a three-dimensional cone was formed in the parameter space (Figure 2).

The article "Stereotactic Surgery of Parkinson's Disease with Magnetic Resonance Imaging under Three-Dimensional Mark Point Positioning Algorithm" was published in 2022. Journal: Contrast Media Mol Imaging.

On the basis of positioning of the center of the circular mark points, the flow of mark point positioning and matching is shown in Figure 3. First, the coordinate position of point AB was determined, and the collinearity of multiple points was found. The mark point module utilized one-mark point matching module in the image acquisition channel, which matched the mark points in a certain order.

### 2.4. Surgical Operating Methods

Surgical target positioning was carried out in the control group. After the CRW stereotaxic head coil was installed, MRI scanning was performed in the sagittal, transverse, and coronal planes. The target was determined by the image direct positioning method combined with coordinate value positioning, and the target coordinates were calculated. As the microelectrodes and electrophysiological recording system produced by FHC Inc. were used, the functional positioning of the anatomically positioned targets was made and confirmed.

In the observation group, stereotaxic surgery and MRI anatomical positioning were given. The puncture path was designed to avoid the cerebral ventricles and cerebral sulcus blood vessels as much as possible. Before surgery, the scalp incision was cut according to the designed puncture path under local anesthesia, the skull was drilled, and the puncture was performed through the bone hole. The hard channel of the puncture sleeve was indwelled, the recording electrode was implanted at the target coordinates through the puncture sleeve, and the discharges of neurons in different positions were recorded. Satisfactory subthalamic nucleus (STN) and substantia nigra spontaneous discharge signals were obtained, which showed high-frequency and high-amplitude cell discharges with high background noise and tremor-related cells. Electrophysiological recording of STN targets was made, eliminating the influence of image drift and brain tissue displacement caused by intraoperative cerebrospinal fluid loss. After the position of the target point was determined, the stimulating electrode was implanted, and the discharge stimulation was conducted while the patient kept awake. The self-reported symptoms and symptom changes of the patients after the electrical stimulation were recorded under electrical stimulations in different frequencies and amplitudes, for the setting and adjustment of the electrical stimulation parameters in the later stage. The initial stimulation parameters were generally set to a frequency of 130 Hz, a pulse width of 60 *μ*s, and a voltage of 1.0–1.5 V. The stimulation voltage was adjusted according to the patient's tolerance and response, generally not exceeding 3.0 V. As the recording was completed, the stimulation was stopped, and the stimulating electrode was fixed. MRI was performed for checking and verifying the position of electrode implantation, and it was observed whether the intracranial hemorrhage or other complications occurred. Afterwards, general anesthesia was given. A saccular space was freed subcutaneously of the right chest, and the stimulation pulser was embedded. The subcutaneous tunnel from the right chest incision to the cephalic incision was connected and penetrated, and the connecting wire was embedded to connect the stimulating electrode and the stimulation pulser. The program controller was used in vitro for detecting the connection of the deep brain stimulation system. After the connection was detected to work normally, the system was shut down temporarily, and the incisions were sutured. Levodopa drugs were retaken in the preoperative dose after surgery. The cerebral edema subsided, and the microdamage effect disappeared 1 month after surgery.

The article "Stereotactic Surgery of Parkinson's Disease with Magnetic Resonance Imaging under Three-Dimensional Mark Point Positioning Algorithm" was published in 2022. Journal: Contrast Media Mol Imaging.

The curative effect of PD patients was judged depending on their emotional state, mental state, and behavior pattern. The side effects of drugs, motor function, activities of daily living, and so forth were also evaluated. Patients' status was assessed 1 month before surgery and 1 month after surgery, respectively; the dose of medication remained unchanged after surgery. With the equation preoperative UPDR−postoperative UPDRS/preoperative UPDRS × 100%, it was evaluated whether the symptoms were improved.

### 2.5. Image Processing

Noise would reduce the signal-to-noise ratio of the image, in which edge detection cannot be performed well. This affects the accuracy and speed of marking seriously. Therefore, it is necessary to denoise the obtained images. Noise interference must be avoided before the mark point positioning, and the identification of mark points was needed after edge detection. The wavelet change was developed by the Fourier transform, with the square integrated in the real number domain of the signal *W*. The Fourier change was $\hat{W}$, *W*, and $\hat{W}$, which can decay fast enough. Then, the function equation was generated.

(1) $$\begin{array}{c} ab\left(w\right)\frac{1}{\sqrt{a}}\left(\frac{tb}{a}\right). \end{array}$$

In equation (1), *b* was the translation factor and *a* was the expansion factor. After the wavelet was established and satisfied, the continuous integrable function *f*(*W*) in the real number domain was expressed as the following equation:

(2) $$\begin{array}{c} f\left(w\right)=\frac{1}{c}\frac{1}{a^{2}}wf\left(a,b\right)\left(\frac{tb}{a}\right)\text{d}a\text{d}b. \end{array}$$

The article "Stereotactic Surgery of Parkinson's Disease with Magnetic Resonance Imaging under Three-Dimensional Mark Point Positioning Algorithm" was published in 2022. Journal: Contrast Media Mol Imaging.

### 2.6. Statistical Analysis

SPSS19.0 was used for statistical analysis of the data in this study. The measurement data was expressed in the form of mean ± standard deviation, and the nonconforming enumeration data were expressed in the frequency (%). *t*-test was adopted to compare differences in the data, and *P* < 0.05 indicated that the difference was statistically significant.

## 3. Results and Analysis

### 3.1. Preprocessing of MRI Images

The results of brain MRI imaging analysis showed that after the image was denoised, Figure 4(b) had a higher clarity than Figure 4(a). Noise reduced the signal-to-noise ratio of the image. After denoise, the mark points in the image could be clear positioned, and edge detection could also be performed for mark point recognition.

### 3.2. MRI Image under Three-Dimensional Mark Point Positioning Algorithm

MRI of PD patients was evaluated, and the results are shown in Figure 5. Figures 5(a)–5(c) clearly show the brain structure as well as the diseased location of the PD patient in different axial positions. Figures 5(d)–5(f) are the effect diagrams using three-dimensional mark point positioning to process the MRI images in different axial positions. It could be observed that it realized the positioning of the diseased location of the patient.

### 3.3. Positioning Effect of MRI Images

For the MRI images of patients in the observation group, the correlation coefficient distribution within the XYZ axes of the anatomical points is shown in Figure 6. The anatomical points were distributed within the patients with a correlation coefficient ≥0.9, and the correlation coefficient between the *Y* axis and the *Z* axis was also ≥0.9. It suggested that the repeatability was very high, and the stability was great.

Eight three-dimensional mark points in the brain MRI image were selected, respectively, with the same positioning accuracy and the same Talairach grid system of each set of data. The transformation parameters of the global registration were also the same.  Figure 7 shows that, for the main body classification of lateral brain and lateral ventricle, the positioning mark point 55 had a large error.

The positioning errors of different mark points were selected in the clinical data and the Brain web data set. The statistical results of the positioning errors of different mark point models are shown in Figure 8. The mark point models had a small effect on the accuracy of the mark points in this study.

The article "Stereotactic Surgery of Parkinson's Disease with Magnetic Resonance Imaging under Three-Dimensional Mark Point Positioning Algorithm" was published in 2022. Journal: Contrast Media Mol Imaging.

### 3.4. Evaluation and Comparison of UPDRS for Patients before and after Surgery

The curative effect of patients was counted with the data one month after surgery. The UPDRS evaluation results of patients in the two groups before and after single-target surgery are shown in Figure 9. The curative effect of the two groups after surgery was significantly different from that before surgery, and the difference was significant (*P* < 0.05). The overall curative effect of the observation group was significantly better than that of the control group. The long-term effect was still to be observed in the follow-up.

### 3.5. Comparison of the Curative Effects

As shown in Table 1, 37 cases in the observation group had the markedly effective effect, accounting for 92.5% of all the PD patients in the observation group. 1 case showed the ineffective effect and 2 cases showed the improved effect, accounting for 2.5% and 5%, respectively. In the control group, 35 cases had markedly effective effect, 2 cases went with ineffective effect, and 3 cases were improved, which accounted for 87.5%, 5%, and 7.5%, respectively. The overall curative effect of patients in the observation group was significantly different from that in the control group (*P* < 0.05).

## 4. Discussion

PD cannot be completely cured, and it progresses slowly. Stereotactic surgery has become a fixed surgical method for the treatment of PD, having a significant effect on eliminating tremor and tetany. Chronic electrical stimulation to deep brain, gene therapy, brain core damage, and nerve tissue transplantation are all surgical treatments [20]. Li et al. [21] used a machine learning method of spatial coupling penalty to analyze the MRI images of PD patients and found that MRI images can well identify the ROI of PD patients. Intracranial responses in patients may predict outcomes. Kotecha et al. [22] demonstrated that stereotactic radiosurgery can be very good for the treatment of brain metastases. PD cannot be cured under any surgical treatment, so a surgery is aimed to relieve the condition of patients and improve symptoms, thereby the course of disease would be prolonged and the pain of patients would be reduced. Therefore, not all patients are suitable for stereotactic surgery, which is also the reason why the surgical result cannot reach 100% in a lot of research. Many factors in the surgical treatment play a corresponding role in the diagnosis and treatment of the disease, including the patients' condition, degree of cooperation, clinical experience, and general function status; the selection of the target during the surgery depends on clinical experience of the physicians [23]. Furlanetti et al. [24] experimented with stereotaxic imaging to reduce the duration and cost of image acquisition without compromising accuracy. In this study, 37 patients (92.5%) in stereotactic surgery had an effect markedly effective. Some scholars stated that stereotactic surgery has contraindications for patients over 70 years old, but the age is not a decisive factor. In this study, there is a 71-year-old male patient who underwent the bilateral surgery, and it also showed a good result after surgery. In stereotactic surgery, the installation of the stereotactic instrument should be standard and adjusted to the best position that the patients felt the most comfortable. During the surgery, fixed personnel were selected for projection to ensure the surgery went smoothly. The treatment of PD in China has been carried out with deep brain stimulation surgery, which is nondestructive with relatively few side effects and complications. The curative effect of stereotactic surgery has been affirmed in many studies. This study also proved the effectiveness of the surgery. It costs less and is suitable for promotion at the grassroots level.

The article "Stereotactic Surgery of Parkinson's Disease with Magnetic Resonance Imaging under Three-Dimensional Mark Point Positioning Algorithm" was published in 2022. Journal: Contrast Media Mol Imaging.

MRI can perform imaging in multiple planes, without radiation, and the soft tissue resolution in the images is good. It has shown good results in stereotactic surgery. Functional MRI analyzes the entire brain area from the perspective of functional integration, determines the directionality among brain areas, and connects the brain areas of interest in the model. In this process, it is affected by functional imaging and neuroanatomy, and the “seed point” is generally chosen for functional connection analysis method to discuss the functional connection of PD patients or normal brains in the resting state [25, 26]. Ryman and Poston [27] used biomarkers to explore the neuropathology of PD patients, and the functional characteristics of dopamine in the brain were shown through MRI image analysis. The results of this study showed that MRI had the clear images and high resolution, giving a high accuracy for PD imaging. In stereotactic surgery, 37 cases were treated as markedly effective, accounting for 92.5%. The three-dimensional mark point positioning algorithm was of important clinical significance in MRI imaging of PD patients.

## 5. Conclusion

In this study, the three-dimensional mark point positioning algorithm was applied to the MRI of PD patients, which improved the efficiency of image feature extraction and classification of patients effectively. It was suggested that MRI was significantly improved with a markedly effective rate of 92.5% in stereotactic surgery. Although the mark point positioning algorithm had good results, it cannot achieve 100% in accurate positioning with unavoidable errors. In practical applications, there were still shortcomings such as the inability of test data to completely eliminate the interference of subjective factors, so the indicators can be standardized in further research. As the images selected in this study were relatively single, image anatomical points can be analyzed from multiple angles in the future, and more samples can also be added to expand the study of PD patients.

The article "Stereotactic Surgery of Parkinson's Disease with Magnetic Resonance Imaging under Three-Dimensional Mark Point Positioning Algorithm" was published in 2022. Journal: Contrast Media Mol Imaging.

## Figures and Tables

**Figure 1:** Representation of the same straight line in the parameter space of the image space domain.

**Figure 2:** Schematic diagram of duality in image space and parameter space.

**Figure 3:** Flowchart of mark point matching.

**Figure 4:** Comparison of image denoise processing.

**Figure 5:** MRI images under the three-dimensional mark point positioning algorithm.

**Figure 6:** Correlation coefficient distribution within the XYZ axes in the observation group. ABC indicates different anatomical points.

**Figure 7:** Analysis results of the positioning error of each step for the mark points in the data set.

**Figure 8:** Statistical results of positioning errors of different mark point models.

**Figure 9:** The ability of MRI to diagnose the depth of myometrial invasion. The symbol # indicates the significant difference between the two groups before and surgery (*P* < 0.05) and *∗* indicates that before surgery and after surgery in the same group (*P* < 0.05).

**Table 1:** Comparison of curative effects in the two groups.

Groups	Markedlyeffective		Ineffective		Improved	
Observation group	37	92.5%	1	2.5%	2	5.0%
Control group	35	87.5%	2	5.0%	3	7.5%
Chi-square	7.939					
*P* value	0.001					

## Data Availability

The data used to support the findings of this study are available from the corresponding author upon request.
